# Mineralocorticoid Receptor Signaling as a Therapeutic Target for Renal and Cardiac Fibrosis

**DOI:** 10.3389/fphar.2017.00313

**Published:** 2017-05-29

**Authors:** Greg H. Tesch, Morag J. Young

**Affiliations:** ^1^Department of Nephrology, Monash Health, ClaytonVIC, Australia; ^2^Monash University Department of Medicine, Monash Health, ClaytonVIC, Australia; ^3^Centre for Inflammatory Diseases, Monash Health, ClaytonVIC, Australia; ^4^Hudson Institute of Medical Research, ClaytonVIC, Australia

**Keywords:** mineralocorticoid receptor, aldosterone, kidney, cardiac, fibrosis

## Abstract

Activation of the mineralocorticoid receptor (MR) plays important roles in both physiological and pathological events. Blockade of MR signaling with MR antagonists (MRAs) has been used clinically to treat kidney and cardiac disease associated with hypertension and other chronic diseases, resulting in suppression of fibrosis in these organs. However, the current use of steroidal MRAs has been limited by off target effects on other hormone receptors or adverse effects on kidney tubular function. In this review, we summarize recent insights into the profibrotic roles of MR signaling in kidney and cardiovascular disease. We review experimental *in vitro* data identifying the pathological mechanisms associated with MR signaling in cell types found in the kidney (mesangial cells, podocytes, tubular cells, macrophages, interstitial fibroblasts) and heart (cardiomyocytes, endothelial cells, vascular smooth muscle cells, macrophages). In addition, we demonstrate the *in vivo* importance of MR signaling in specific kidney and cardiac cell types by reporting the outcomes of cell type selective MR gene deletion in animal models of kidney and cardiac disease and comparing these findings to those obtained with MRAs treatment. This review also includes a discussion of the potential benefits of novel non-steroidal MRAs for targeting kidney and cardiac fibrosis compared to existing steroidal MRAs, as well as the possibility of novel combination therapies and cell selective delivery of MRAs.

## Introduction

The mineralocorticoid receptor (MR) is a ligand activated cytosolic receptor that has received increasing attention as a driver of cardiovascular and renal fibrosis. Although best known as an “aldosterone receptor” that regulates electrolyte and fluid homeostasis in the distal nephron and other epithelial tissues, the MR is expressed widely at low levels in the cardiovascular system, in podocytes and other kidney cells, central nervous system and adipocytes among others. While the primary mineralocorticoid ligand for the MR is aldosterone, the MR can also bind and respond to glucocorticoids; ligand selectivity for the MR in mineralocorticoid target tissues, including renal epithelial cells, colon, discrete nuclei in the brain, and the vessel wall, is thus maintained by pre-receptor metabolism of glucocorticoids by the enzyme 11β-hydroxysteroid dehydrogenase type 2 (HSD2) (Chapman et al., 2013). In many tissues including cardiomyocytes, immune cells, and adipocytes, HSD2 is absent and cortisol/corticosterone, which circulate at higher levels than aldosterone, can bind and regulate the receptor.

A role for the MR in fibrosis was proposed by Brilla and Weber (1992) in studies demonstrating profibrotic effects of aldosterone infusion in high salt fed rats. The studies echoes the much earlier work of Selye (1958), who described granulomatous tissue and fibrosis in peripheral organs in dogs given high doses of the mineralocorticoid deoxycorticosterone (DOC), although it was thought to be a glucocorticoid effect at the time. The work of Brilla and Weber and other labs lead to the Randomized ALdactone Evaluation Study (RALES; Pitt et al., 1999), which formally demonstrated the therapeutic protective effects of spironolactone in all cause heart failure. However, the risk of hyperkalemia with the clinical use of MR blockers has limited their use. This review will discuss tissue and cell specific aspects of MR signaling in fibrosis of the kidney and heart and the potential strategies for better targeting MR in fibrotic disease.

## MR Signaling in Kidney Fibrosis

### Aldosterone and Chronic Kidney Disease

Glomerular and interstitial fibrosis are features of chronic kidney disease (CKD) which, if allowed to progress, can result in the development of end-stage renal failure and patients requiring renal replacement therapy (kidney transplantation or dialysis) to survive. CKD is associated with an adverse rise in circulating aldosterone levels with respect to extracellular volume, which increases as glomerular filtration rate falls. This state of relative hyperaldosteronism leads to activation of the MR in kidney cells which can facilitate proinflammatory and profibrotic responses, particularly in non-epithelial cells (Schwenk et al., 2015). Therefore, aldosterone-induced MR signaling may be a key factor in promoting fibrosis in CKD. Furthermore, current standard of care therapy for CKD, which involves blockade of the renin–angiotensin system (RAS) by angiotensin-converting enzyme inhibitors (ACEi) or angiotensin receptor blockers (ARBs), will cause a paradoxical rise in aldosterone in 30–50% of patients, often referred to as “aldosterone breakthrough” (Schwenk et al., 2015). Hence, there is an important need to inhibit MR signaling in CKD.

### Use of Mineralocorticoid Receptor Antagonists in Chronic Kidney Disease

Clinical trials have shown that MR antagonists (MRAs), including spironolactone (a first generation non-selective steroidal MRA), eplerenone (a second generation selective steroidal MRA) and finerenone (a third generation selective non-steroidal MRA) are all capable of providing protection against CKD. So far, most of these studies have involved the addition of spironolactone to RAS blockade with an ACEi or ARB. In diabetic nephropathy patients, spironolactone provides additional suppression of albuminuria compared to RAS blockade alone, and this protection appears to be partly independent of any effect on blood pressure (Guney et al., 2009; Mehdi et al., 2009; Esteghamati et al., 2013). Similar findings have been found in patients with albuminuria resulting from non-diabetic CKD (Furumatsu et al., 2008; Tylicki et al., 2008; Bianchi et al., 2010). Further analysis has shown that the protective effects of spironolactone are associated with reductions in the urine levels of transforming growth factor β TGF-β1 (Guney et al., 2009), collagen IV (Furumatsu et al., 2008), and amino-terminal propeptide of type III procollagen (Tylicki et al., 2008), suggesting that spironolactone is inhibiting renal fibrosis in these patients.

Clinical studies have also demonstrated that the addition of eplerenone or finerenone to RAS blockade provides greater suppression of albuminuria in patients with diabetic nephropathy (Epstein et al., 2006; Bakris et al., 2015) and non-diabetic CKD (Boesby et al., 2011). However, the specific effects of MRAs on renal fibrosis were not assessed in these studies.

Despite these benefits, the use of MRAs in CKD has drawbacks which can limit its clinical use. For example, spironolactone also binds to progesterone and androgen receptors which can lead to adverse progestational and anti-androgenic effects (Danjuma et al., 2014). In comparison, eplerenone is more selective, but has weaker affinity for binding MR and is less potent than spironolactone. A further downside of MRA therapy is that it can cause hyperkalemia in patients, which is a major clinical concern, particularly in the context of renal impairment, and necessitates withdrawal of this treatment (Mehdi et al., 2009; Bianchi et al., 2010; Esteghamati et al., 2013). This problem arises because MRAs inhibit the activation of ion channels in tubule cells by aldosterone, which is required for maintaining sodium and potassium homeostasis. Blocking this pathway elevates potassium levels, which is exacerbated during RAS blockade. However, recent preclinical and early phase clinical trial evidence suggests that this problem may be reduced using finerenone (a non-steroidal MRA) which can inhibit pathological MR signaling as effectively as spironolactone while having a minimal effect on potassium homeostasis (Bakris et al., 2015). A potential explanation for the lack of effect of finerenone on potassium levels has been identified by radioactive labeling studies showing that finerenone is almost equally distributed in heart and kidney which contrasts with steroidal MRAs (spironolactone and eplerenone) which show greater accumulation in the kidney (Kolkhof et al., 2014). This suggests that the protective effects of MR blockade in heart and kidney can be achieved with finerenone at a dose that has reduced risk of hyperkalemia, which is proposed to be due to structural differences that influence its selective uptake in target tissues.

### Effects of Mineralocorticoid Receptor Antagonists in Animal Models of Renal Fibrosis

The anti-proteinuric effects of MRAs have also been seen in a variety of animal models of CKD, including diabetic nephropathy, hypertensive nephropathy, lupus nephritis, polycystic kidney disease, and cyclosporine A nephrotoxicity, which in some cases are also associated with protection of renal function (Guo et al., 2006; Monrad et al., 2008; Nemeth et al., 2009; Miana et al., 2011; Jeewandara et al., 2015; Sun et al., 2015). In models of diabetic nephropathy and hypertensive nephropathy, MRAs have been shown to provide additional protection when combined with an ACEi, compared to either therapy alone, and their benefit is often independent of an effect on blood pressure (Kang et al., 2009; Nemeth et al., 2009; Zhou et al., 2016).

Analysis of tissues from acute and chronic animal models of kidney disease have shown that MRAs suppress the development of glomerulosclerosis and interstitial fibrosis, which is usually linked to reduced production or deposition of matrix proteins (e.g., collagen, fibronectin) and profibrotic molecules (e.g., TGF-β1, plasminogen activator inhibitor-1 [PAI-1], connective tissue growth factor [CTGF]) (Trachtman et al., 2004; Kang et al., 2009; Sun et al., 2015). In addition, MR blockade in these models can reduce podocyte injury (Nemeth et al., 2009), autoantibodies (Monrad et al., 2008), kidney leukocyte accumulation (Guo et al., 2006; Huang et al., 2014), and expression of molecules which drive inflammation (e.g., monocyte chemoattractant protein-1 [MCP-1], tumor necrosis factor [TNF]-α) (Huang et al., 2014; Zhou et al., 2016), suggesting that the anti-fibrotic effects of MRAs may, in part, arise indirectly from the inhibition of inflammation and apoptosis in the kidney.

### Infusion of MR Ligands Promotes Renal Injury and Fibrosis in Rodents

Prolonged aldosterone infusion into rats and mice results in a model of hyperaldosteronism which causes hypertension, podocyte injury, kidney inflammation, proteinuria, and renal fibrosis (Blasi et al., 2003). This renal injury and fibrosis can be blocked with MRA treatment and is reduced in mice lacking galectin-3 (Calvier et al., 2015), PAI-1 (Ma et al., 2006), interleukin-18 (IL-18) (Tanino et al., 2016), or inflammasome activation in macrophages (Kadoya et al., 2015), suggesting their involvement in the MR-mediated renal fibrosis.

Studies have also shown that infusion of hydrocortisone or angiotensin II (AngII) can induce renal injury in aldosterone deficient rodents, which is inhibited by MRAs (Rafiq et al., 2011; Luther et al., 2012). This suggests that cortisol (an MR ligand) and AngII (via binding to its receptor) may also activate MR to cause renal injury. The potential for cortisol to activate MR is particularly high in kidney macrophages which, unlike most other kidney cells, lack HSD2 that normally converts cortisol to a metabolite that is incapable of activating MR (Brown, 2013).

### Aldosterone Induces Fibrotic Responses in Kidney Cells

Aldosterone can directly promote fibrotic responses in cultured kidney cells. For example, aldosterone stimulates proliferation of mesangial cells and kidney fibroblasts via transactivation of epidermal growth factor receptor (EGFR), platelet-derived growth factor receptor (PDGFR) (Huang et al., 2009, 2012). Aldosterone can also induce myofibroblastic transdifferentiation in mesangial cells and tubular epithelial cells (Zhang et al., 2007; Diah et al., 2008). In addition, aldosterone can directly stimulate the gene expression and synthesis of profibrotic cytokines (TGF-β1, PAI-1, CTGF; Huang et al., 2008; Terada et al., 2012) and matrix proteins (fibronectin and collagens; Nagai et al., 2005; Lai et al., 2006; Diah et al., 2008; Chen et al., 2013) in mesangial cells and kidney fibroblasts. These responses were shown to be dependent on the generation of reactive oxygen species and signaling via Rho-kinase, phosphoinositide 3-kinase (PI3K), extracellular signal-regulated kinase 1/2 (ERK1/2), c-jun N-terminal kinase (JNK), or small body size mothers against decapentaplegic-2 (SMAD2).

### Lessons from MR Deletion in Specific Cell Types in Models of Kidney Disease

The specific roles of MR in some cell types (macrophages, podocytes, vascular smooth muscle cells, and endothelial cells) have been examined in models of kidney disease in transgenic mice where MR is selectively deleted in these cells. Studies have shown that deficiency of endothelial MR has no effect on renal injury induced by DOC acetate/salt (Lother et al., 2016) and deficiency of podocyte MR has no effect on the development of anti-glomerular basement membrane (anti-GBM) glomerulonephritis (Huang et al., 2014). In contrast, deficiency of MR in smooth muscle cells has recently been shown to limit ischemia-reperfusion injury in the kidney through effects on Rac1-mediated MR signaling (Barrera-Chimal et al., 2017). Remarkably, deficiency of MR in macrophages was found to have similar protection to eplerenone treatment in a model of anti-GBM glomerulonephritis (Huang et al., 2014). This suggests that macrophage MR signaling may be the major cause of MR-mediated injury in CKD driven by macrophage-dependent inflammation, which include progressive forms of glomerulonephritis and diabetic nephropathy.

## MR Signaling in Cardiac Fibrosis and Heart Failure

### A Role for MR Signaling in Heart Failure

Heart failure is defined as failure of the pump function of the myocardium and is caused by many factors including structural remodeling of the ventricle wall due to myocardial hypertrophy and elevated interstitial fibrosis. Cardiac fibrosis, due to increased deposition and crosslinking of extracellular matrix (ECM) proteins, results in increased stiffness of the tissue, which leads to poor ventricular relaxation and reduced contractile force (Travers et al., 2016). Together with “remodeling” of ion channel function and other cellular pathways (Cohn et al., 2000) these functional changes limit cardiac output, underpinning the transition from compensated to decompensated cardiac hypertrophy. Many signaling systems contribute to the development of cardiac pathological changes including increased activation of the MR.

As noted above, the RALES and other clinical trials investigated the benefits for MRA as add on therapy to current best practice therapy and demonstrated a role for MR signaling in all-cause heart failure, heart failure post-MI and in mild heart failure (Pitt et al., 1999, 2003; Zannad et al., 2010). These trials validated many preclinical studies of cardiovascular disease (CVD), as well as the renovascular disease models discussed above, that showed equivalent protection for MRA—spironolactone and eplerenone—in a range of rodent models of cardiac fibrosis including aldosterone or DOC infusion plus salt, elevated AngII, low nitric oxide (N-nitro-L-arginine methyl ester [L-NAME]), pressure overload (transverse aortic constriction [TAC]), myocardial infarction (MI), spontaneously hypertensive rats and Dahl salt-sensitive rats (Young, 1995; Rocha and Funder, 2002; Oestreicher et al., 2003; Mihailidou et al., 2009; Lother et al., 2011). Moreover, it has also been demonstrated using subpressor doses of MRA or central administration of MRA to block hypertension that MR-mediated cardiac fibrosis is independent of blood pressure changes (Bauersachs and Fraccarollo, 2003). Together these studies underscore the importance of MR signaling, directly in the heart, for disease settings in which tissue injury, oxidative stress, and inflammation are common factors. Thus, MRA likely exert cardio-protective effects via direct blockade of cardiac and vascular MR.

### Mechanisms of MR-Mediated Cardiac Fibrosis

The diffuse interstitial and perivascular collagen depots that characterize established cardiac fibrosis are preceded by early tissue injury and inflammation responses that can be detected within days of MR activation (Young et al., 2003; Wilson et al., 2009). Similar to the kidney, MR activation promotes oxidative stress in the vessel wall and the expression of inflammatory factors including chemoattractant proteins (MCP-1/chemokine (C-C motif) ligand 2 [CCL2], chemokine (C-X3-C motif) ligand 1 [CX3CL1], chemokine (C-C motif) ligand 5 [CCL5], etc.) and adhesion molecules (intercellular adhesion molecule-1 [ICAM-1], vascular cell adhesion molecule-1 [VCAM-1]) that facilitate the recruitment of inflammatory cells to the myocardium (Fuller and Young, 2005). Activated tissue macrophages and T-cells release proinflammatory cytokines (TNF-α, inducible nitric oxide synthase [iNOS], osteopontin, etc.) to amplify type-1 proinflammatory responses in the tissue (Travers et al., 2016). Resolution of the inflammatory response and the transition to anti-inflammatory and repair phenotypes is essential to maintain normal myocardial function and involves expression of common trophic and profibrotic factors such as TGF-β, platelet-derived growth factor (PDGF), CTGF, and PAI-1 among others (Rickard and Young, 2009; Shen et al., 2016). Studies have also shown that oxidative stress in cardiomyocytes can induce MR activation in a Rac1-dependent, ligand-independent manner, and thereby promote cardiac injury (Nagase et al., 2012; Ayuzawa et al., 2016). In addition, cardiac overexpression of constitutively activated Rac1 promotes MR activation and cardiac fibrosis (Lavall et al., 2017). Elevated fibrosis is essential for the resolution of major insults such as MI in which reparative scar tissue is absolutely required to replace necrotic myocytes and maintain ventricle wall integrity. In contrast, reactive fibrosis in viable tissue in response to MR signaling only serves to limits cardiac function and is the focus of considerable efforts to identify therapeutic targets (Fraccarollo et al., 2011).

### Experimental Models for MR-Dependent Cardiac Fibrosis

Mice with MR deficiency in specific cell types have been used to determine cell-selective MR signaling mechanisms in cardiac fibrosis. As noted above, the macrophage was identified as a novel site of MR signaling in cardiac remodeling; loss of macrophage MR signaling had a profound protective effect in terms of tissue inflammation and fibrosis, despite little or no changes in the recruitment of macrophages in some models (Rickard et al., 2009; Usher et al., 2010; Bienvenu et al., 2012). Specifically, mice lacking MR in macrophages are protected from DOC/salt and L-NAME/AngII mediated cardiac inflammation and fibrosis and most recently, atherosclerosis (Rickard et al., 2009; Bienvenu et al., 2012). The type 1 proinflammatory response is markedly reduced in these models as are pro-repair/pro-fibrotic signals and the expression of α-smooth muscle actin (α-SMA) expressing fibroblasts in the myocardium (Shen et al., 2016). In trying to explain this outcome, other investigators have suggested that the MR null macrophage has an M2 like phenotype, which may be immunomodulatory and limit tissue remodeling (Usher et al., 2010). In addition, evidence from different groups support a role for MR signaling in promoting an M1 proinflammatory phenotype in macrophages (Rickard et al., 2009; Martin-Fernandez et al., 2016). To this end, recent efforts to determine the cell signaling pathways regulated by MR signaling suggest that proinflammatory signaling via JNK/activating protein-1 (AP-1), and potentially nuclear factor-kappa B (NF-κB)/p65, transactivation pathways are MR-dependent (Shen et al., 2016; Sun et al., 2016). The MR is also involved in direct gene transcriptional responses in the macrophage, including for MR target genes such as p22phox, PAI-1 (Calo et al., 2004). Consistent with studies of transcriptional regulation of macrophages the overall effect of MR activation is most likely dependent upon macrophage phenotype (Barish et al., 2005). Taken together, these knockout studies validate the importance of macrophages and early inflammation in promoting the overall fibrotic response. However, MR signaling elsewhere in the cardiovascular system is also important.

Deletion of the MR from cardiomyocytes is sufficient to block reactive, but not reparative fibrosis in the heart. In a model of MI, cardiomyocyte MR null mice demonstrated improved reparative scar formation in the infarcted zone, increased revascularization of the tissue and improved cardiac function, but reduced reactive fibrosis in the viable ventricle wall (Fraccarollo et al., 2011). The improved remodeling profile was associated with lower inflammatory and profibrotic marker expression but more importantly, these data demonstrated a dual role for cardiomyocyte MR in the cardiac tissue response to an ischemic event that was highly dependent upon the tissue context. In support of these data, studies investigating the DOC/salt reactive fibrosis model and the TAC model showed that, whereas DOC/salt-mediated tissue inflammation and fibrosis were prevented in cardiomyocyte MR null mice (Rickard et al., 2012), pressure-overloaded hearts were not similarly protected (Lother et al., 2011). Despite these differences in tissue remodeling, cardiac function in each of the disease models was universally improved in hearts in which MR signaling was absent, indicating a separation of MR signaling effects in the heart. We also detected up-regulation of antifibrotic mechanisms including enhanced expression of ECM protein decorin, which can block TGF-β and CTGF (Rickard et al., 2012). These data support earlier studies showing elevated aldosterone levels can block antifibrotic pathways.

MR in the endothelial cell and vascular smooth muscle cell (VSMC) layers of the vessel wall regulate important aspects of vascular physiology. Contractile and relaxation responses are MR-dependent and require MR signaling in both cells types, whereas cell-selective deletion studies of the MR shows that VSMC MR but not endothelial cell MR are required for age-related and other forms of hypertension (McCurley and Jaffe, 2012; Rickard et al., 2014). In fact, endothelial cell MR deficiency had negative effects on nitric oxide production and signaling that resulted in aberrant vascular functional responses in unchallenged tissues (Jaffe and Jaisser, 2014; Rickard et al., 2014). However, endothelial cell MR null mice are protected from cardiac inflammation and fibrosis induced by exogenous mineralocorticoids and cardiovascular remodeling and dysfunction due to diet-induced obesity (Schafer et al., 2013; Rickard et al., 2014; Jia et al., 2016). Although adhesion molecules such as ICAM-1 can be directly regulated by aldosterone/MR signaling in endothelial cells (Caprio et al., 2008), studies now suggest it may not be the primary regulator of MR-mediated fibrosis (Salvador et al., 2016). In contrast, recent work by Marzolla et al. (2017) has identified enhanced atherosclerotic plaques in aldosterone-treated ApoE^-/-^ mice and has shown that macrophage recruitment in these lesions is dependent on MR-mediated ICAM-1 signaling and that ICAM-1 is directly regulated by MR in HUVEC cells. The complexity of the endothelial MR signaling was further demonstrated by research which validated its role in DOC/salt mediated cardiac fibrosis but not renal fibrosis, suggesting interaction with permissive signaling factors that are specific to organs or vascular bed (Lother et al., 2016).

MR signaling in VSMC can also regulate tissue fibrosis, either as fibrosis of the vessel wall and perivascular space or via facilitating inflammatory cell influx and activation. We and others have shown vascular inflammation and oxidative stress to precede the onset of aldosterone-mediated cardiac fibrosis (Rocha and Funder, 2002; Wilson et al., 2009; McCurley and Jaffe, 2012). This in turn promotes endothelial cell damage which further enhances oxidative stress and inflammation leading to uncoupling of endothelial nitric oxide synthase (eNOS), production of peroxynitrate species and further potentiation of vessel wall injury and the recruitment of monocytes and macrophages to the surrounding tissue. In addition to the important role of VSMC MR in blood pressure control, MR also plays a key role in VSMC in the pathological remodeling following MI (Gueret et al., 2016). The authors showed increased left ventricle compliance, preserved coronary vascular reserve and reduced tissue fibrosis in VSMC MR null versus wild type mice subjected to MI. The VSMC is also of interest in MR signaling given the evidence supporting crosstalk between the MR and AngII signaling pathways in pathological processes in cardiovascular tissues, which support the use of MRA as well as AngII signaling blockers for the management of CVD (Jaffe and Mendelsohn, 2005).

### Insights into Pharmacological Targeting of MR in Kidney and Cardiovascular Disease

As noted previously, the first MRA, spironolactone, was succeeded by MR selective eplerenone following the success of the RALES trial to address side effects associated with binding at sex steroid receptors. However, hyperkalemia remained a significant side effect for these MRAs. Several non-steroidal MRAs, which potently and selectively inhibit MR, are now being examined for their impact on cardiac and renal diseases and hyperkalemia, of which finerenone (or BAY-94-8862 from Bayer) is in phase 3 trials for end stage renal failure. Finerenone, CS-3150 (from Daiichi Sankyo) and PF-03882845 (from Pfizer) have been investigated in DOC/salt mediated renal and cardiac fibrosis and other forms of kidney disease and show protective effects that are equivalent to eplerenone. The development of MRAs has recently been reviewed in detail (Kolkhof et al., 2016).

Recent insights into the mechanisms of MR-dependent fibrosis has raised the possibility of combining MRAs (at a dose that avoids hyperkalemia) with other therapies that target the downstream effects of MR signaling in order to minimize organ injury. Given that oxidative stress and MAPK signaling are important for mediating the profibrotic effects of MR signaling in the kidney and heart (**Figure 1**), it is likely that therapies which specifically target these mechanisms, if well tolerated, could be used in conjunction with MRAs to provide better suppression of MR-dependent fibrosis. In addition, there are other novel therapies which attenuate models of MR-mediated cardiac fibrosis, including the insulin sensitizing drug Metformin (Mummidi et al., 2016), antagonism of chemokine receptor (C-X-C motif) receptor 4 (CXCR4) (Chu et al., 2011) and treatment with a high fiber diet to enhance healthy gut microbiota (Marques et al., 2017). These therapies offer novel insights into the mechanisms of disease and could also be combined with MRAs or other injury-suppressing drugs to reduce fibrotic disease.

**FIGURE 1:** Proposed mechanisms of MR-mediated fibrosis in the kidney and heart. MR ligands (Aldo, aldosterone; Cort, cortisol) bind with cytoplasmic MR resulting in: (i) translocation of the MR to the nucleus and activation of transcription of profibrotic genes (TGF-β1, PAI-1, CTGF, collagens, fibronectin); (ii) induction of oxidative stress in mitochondria resulting in transdifferentiation of epithelial and mesangial cells into a more profibrotic myofibroblast phenotype; (iii) increased nicotinamide adenine dinucleotide phosphate (NADPH) oxidase activity and oxidative stress in macrophages, cardiomyocytes, and podocytes leading to enhanced MR activation (via Rac1) and worsening inflammation and injury which subsequently promote fibrosis; or (iv) transactivation of growth factor receptors, which facilitate oxidative stress, rapid activation of mitogen-activated protein kinase (MAPK) signaling and proliferation of fibroblast-like cells.

Studies involving cell selective deletion of MR in models of kidney and CVD have indicated the potential benefits of selectively delivering MRAs to macrophages, cardiomyocytes, and vascular smooth muscle cells. If MRAs could be selectively delivered to these cells with carriers that recognize cell surface molecules that are restricted to these cell types, then the problem of hyperkalemia could be avoided. Animal studies have shown that drugs can be selectively targeted to macrophages using a variety of nanoparticles (He et al., 2017), however, the development of these delivery systems is in the very early stages and needs further progress.

## Conclusion

Cardiovascular and kidney diseases are a major health problem worldwide, with the incidences becoming more prevalent in an aging population and with the growing epidemic of obesity and type 2 diabetes. Given the critical role of MR signaling in kidney and cardiac fibrosis, effective and selective targeting of the pathological effects of MR signaling in these organs remains a high priority for treatment. Hopefully, this can be achieved with emerging novel MR inhibitors, combination therapies, or cell selective delivery of MRAs, leading to better patient outcomes.

## Author Contributions

GT wrote the section of this review on MR signaling in kidney disease and co-wrote the abstract, introduction, the insights into pharmacological targeting of MR and the conclusion. GT also developed **Figure 1**. MY wrote the section of this review on MR signaling in cardiac disease and co-wrote the abstract, introduction, the insights into pharmacological targeting of MR and the conclusion. Both authors approved of the final revised manuscript.

## Conflict of Interest Statement

The authors declare that the research was conducted in the absence of any commercial or financial relationships that could be construed as a potential conflict of interest.
